# Nexus of green energy, financial inclusion, militarization, and environmental sustainability: A global perspective

This article has been retracted.

**DOI:** 10.1371/journal.pone.0301122

**Published:** 2024-05-17

**Authors:** Muhammad Ramiz Murtaza, Fan Hongzhong, Radulescu Magdalena, Haseeb Javed, Sinisi Crenguta Ileana

**Affiliations:** 1 School of Economics, Huazhong University of Science and Technology, Wuhan, China; 2 Department of Finance, Accounting, and Economics, National University of Science and Technology, Politehnica Bucharest, Pitesti Regional Center, Pitești, Romania; 3 Institute of Doctoral and Post-Doctoral Studies, University Lucian Blaga of Sibiu, Sibiu, Romania; 4 School of Business Administration, Budapest Metropolitan University, Budapest, Hungary; 5 School of Management, Valahia University of Târgoviște, Târgoviște, Romania; 6 Selinus University of Science and Literature, Bolonga, Italy; Second Xiangya Hospital, Central South University, CHINA

## Abstract

This article investigates the dynamic impact of green energy consumption (GE), financial inclusion (FI), and military spending (MS) on environmental sustainability (ES) by utilizing a sample of 121 countries from 2003 to 2022. The dataset is divided into high-income, upper-middle income and low and lower-middle-income countries. We employed a two-step system GMM approach, which was further robust through panel Quantile and Driscoll-Kraay (D-K) regressions. The findings divulged that green energy resources benefit ES at global and all income levels because of having a significant negative impact of 5.9% on ecological footprints. At the same time, FI and MS significantly enhance ecological footprints by 7% and 6.9%, respectively, proving these factors detrimental to ES. Moreover, conflicts (CON), terrorism (TM), institutional quality (IQ), and socioeconomic conditions (SEC) also have a significantly positive association with global ecological footprints and most of the income level groups. Dissimilarly, financial inclusion and armed conflicts have a non-significant influence on ecological footprints in low-income and high-income countries, respectively. Furthermore, institutional quality enhances ES in upper-middle and low and lower-middle-income countries by negatively affecting ecological footprints. At the same time, terrorism significantly reduces ecological footprints in high-income countries. This research also provides the imperative policy inferences to accomplish various SDGs.

## 1. Introduction

Environmental sustainability is a contemporary developmental challenge on the planet, and its impacts proliferate globally and at a basic level [1]. Environmental sustainability (ES) can not be assured if the global environment is poorly harmed, and joint action is needed to counter this matter [2]. According to the Global Footprint Network (GFN), the world’s biocapacity is lesser than the global populace’s ecological footprints, which means that the world is deteriorating the environment more than the absorption capacity of the ecosystem.

As a global action, the United Nations presented 17 sustainable development goals (SDGs), which guide nations around the globe to grow their economies without deteriorating the ecology, and these goals should be achieved by 2030. As an essential requirement for humanoid socioeconomic endeavors, energy is a prominent element for ecological deterioration [3]. Therefore, out of all SDGs, authorities are confronting more enormous challenges regarding SDG-7 & SDG-13, which deal with using green energy and climatic actions correspondingly. These goals push nations around the globe to transform towards green energy consumption for restraining environmental deterioration [4]. Green energy is a combination of skill and technology; therefore, enhancement in the consumption of green energy can endorse ES by reducing all kinds of noxious emissions [5].

A stable financial system can achieve climatic goals by endorsing green innovations in the energy sector [2]. Being an integral chunk of the financial system, financial inclusion develops easy access for businesses and individuals to financial services, including savings, payments, credits, and assurances [6]. These financial aids help firms and individuals in the adoption of green technologies and customs, which consequently favors environmental sustainability [7]. On the other hand, it can harm the environment by enhancing income levels through industrialization and manufacturing [8].

To ensure peace and stability, a significant upsurge in military expenditures has been witnessed, and it has become one of the leading government expenditures around the globe. In the name of national sovereignty, military spending increases more with betterment in the financial system and income levels [9, 10]. An intricate linkage prevails between the environment and human actions. Therefore, several dimensions and factors have been investigated, especially within the recent two decades, ignoring the military as a dimension [1]. A massive amount of energy is required to fulfill military needs, chiefly composed of burning fossil fuels [11]. Moreover, air, water, and the earth’s available biological capacity are collectively damaged by military actions [12]. Fig 1 depicts the overall trend of green energy, military expenditure and various financial inclusion indicators in the selected panel of countries.

**Fig 1:** The overall trend of green energy, financial inclusion, and military expenditure [Source: WDI & IMF].

Recently, the United Nations Framework on Climate Change (UNFCCC) organized the 28^th^ conference of parties (COP-28) in the United Arab Emirates (UAE) with a theme of limiting climatic impact by stopping the use of conventional energy sources. Thus, all the member nations vowed to adopt green energy sources and achieve net zero emissions by 2050. It also highlighted that financial inclusion is mandatory for the green energy transition in all segments of society [13]. Furthermore, Military actions profoundly impact environmental sustainability, and using green energy in this sector can be beneficial for accomplishing climatic goals. Still, researchers ignored it as an environmental determinant [14]. Keeping these recent challenges in view, the prime contribution of this study is to provide an inclusive understanding of achieving environmental sustainability goals by enhancing green energy accessibility through non-discriminate financing and by greening major sectors of the economy, such as the military. Moreover, this research also provides empirical evidence which can assist stakeholders in creating useful framework for mutual co-operation and designing environmental policies to accomplish common climatic goals.

This study analyzes the impact of green energy, financial inclusion, and military on environmental sustainability worldwide in 121 countries and evaluates 44 high-income, 33 upper-middle, and 44 low-and lower-middle-income countries from 2003–2022. To the best of our personal knowledge, no empirical research has been done on a prescribed issue, either on a regional or a transnational level, creating a massive gap for researchers to conduct a global and regional investigation. Fig 2 shows the ultimate relation between concerned factors and ecology.

**Fig 2:** Logical link between the study’s variables.

This research work is unique and influential in various ways. First, this study contributes that the included factors are not just a cause of air pollution; these profoundly influence the sustainability of the whole environment. Hence, ecological footprints are taken as an indicator to denote environmental sustainability because, according to Strezov, Evans [15] and Cui, Weng [16], it has a strong ability to describe environmental sustainability. In addition to carbon emissions, it incorporates other environmental variables (forestry, urbanized land, fishing, grazing, and cropland) to enrich the existing body of knowledge. Second, SDG-7 focuses on the extensive use of green energy around the globe, and according to green theory, it can sustain the economy and environmental quality in the long term. It can play a substantial role in reducing half of the noxious emissions till 2050. Hence, it is decisive to analyze the global potential of green energy to sustain the environment by amalgamating it with momentous socioeconomic factors. Consequently, green energy use is integrated with financial inclusion and the military sector in this study to evaluate the nexus of these variables with ES, which was ignored in prior works. Third, financial inclusion is the access to financial services to individuals and business entities, which can assist in accomplishing various SDGs. Therefore, a comprehensive index of financial inclusion has been generated in this study by incorporating some substantial indicators for better contribution to the prevailing literature and practices.

In addition; the fourth, military is one of the major sectors of each economy around the planet, which refers as a chief consumer of energy, and according to the theory of treadmill of destruction, it has strong negative imprints on the environment. Furthermore, it is also part of SDG-16 because nations spend on the military to ensure peace. Therefore, adopting green energy technologies in this sector can guarantee global environmental sustainability (SDG-13). Thus, military dynamics contribute to this study to achieve global SDGs as there is a prime need to include this sector in environment-related research. Moreover, SDG-16 is substantially linked to all SDGs [17]. Thus, other factors related to SDG-16, such as armed conflicts, terror, and institutional quality, have been included as control factors for unbiased estimation. Fifth, the dataset is divided into three different income level groups: high-income, upper-middle income, and low and lower-middle-income countries for an inclusive contribution to existing literature. Sixth, last but not least, this study provided valuable findings to contribute to the sustainable development theory and policy implications that can assist authorities in accomplishing global SDGs.

Literature about the impact of the military and its dynamics on environmental sustainability is discussed in the next section. The details of data, materials, and methods are given in the third section, while the results of this empirical research are presented in the fourth section. In the last section, results are concluded, and valuable policy recommendations are provided.

## 2. Literature review

A sudden rise in global population and the number of independent nations enhanced the profundity of environmental impacts of human actions. The current generation must sustain environmental quality by discovering ways to nullify damages and enabling our current and future generations to exist on this planet [18]. Out of all other SDGs, environmental sustainability is the primary goal, which focuses on the healthiness of all the components of nature and the preservation of environmental capacity [19]. Researchers are successfully identifying and defining the latest indicators which can intensely affect environmental sustainability [20]. Green energy, financial inclusion, Military spending, wars (armed conflicts), and terrorism are some of the latest indicators of environmental sustainability [21–23]. After closely observing existing literature, the review is presented into variable vice segments to understand better and identify the research gap.

### 2.1. Green energy and environmental sustainability

The advancement of green energy and the impact of its use on environmental sustainability has been the hottest discussion in recent years [24]. It is considered that the usage of green energy profoundly impacts environmental sustainability [25]. In the accumulation of economic benefits, the consumption of green energy can ensure global environmental sustainability by reducing fossil fuel addiction [26].

Employing statistical techniques, taking a different sample, considering dissimilar study periods, and incorporating divergent determinants can generate various results. For example, Cheng, Ren [27] utilized panel quantile regression to analyze the relationship for 6 BRICS nations from 2000 to 2013. They discovered that carbon emissions were reduced due to using green energy. Similar results were found by Charfeddine and Kahia [28] when they employed the panel vector autoregression technique for a panel of 24 MENA countries. In the case of the 15 most clean energy consumer nations, Saidi and Omri [29] discovered that there was no causal association between green energy and carbon emissions in the long run. Still, these variables had causal feedback linkage in the short run. In most recent studies, Adekoya, Ajayi [30] & Grodzicki and Jankiewicz [31] employed ARDL and spatiotemporal approaches for Africa and Europe, respectively. Their studies unveiled that carbon emissions were reduced due to green energy consumption, while economic growth and urbanization proved harmful to environmental sustainability.

Contrarily, Hasnisah, Azlina [32] found that green energy consumption was insignificant in dropping environmental pollution when they investigated the linkage using FMOLS & DOLS techniques for 13 Asian nations.

### 2.2. Financial inclusion and environmental sustainability

Economic growth relies on financial inclusion because it confirms competent resource allocation, capital formation, and investment activities enhancement. In addition to playing a vital role in boosting the economy, the financial sector also ensures environmental sustainability by promoting the use of cleaner energy [26]. Financial inclusion is a genuine representor of accessibility of financial resources from both banks and stock exchanges. It can reduce environmental harm by encouraging investments in the efficiency of the energy sector. Moreover, it also reduces environmental hazards caused by oil use because it stabilizes financing rates [2]. On the other hand, economic activities are increased due to financial inclusion, which is the biggest stake in environmental sustainability [26].

In prior literature, financial development was presented as a financial and economic growth gauge. Financial inclusion is a more effective and latest indicator [33]. In some recent studies, researchers found mixed results after empirically analyzing the association between financial inclusion and environmental sustainability such as Singh, Raza [34] employed quantile regression to investigate the linkage in a panel of G24 nations, and their results disclosed a positive relationship between financial inclusion and ecological footprints. Similar results were found by Ali, Jianguo [33] when they used AMG, PMG, and CCEMG to analyze the linkage for 11 ECOWAS nations. Le, Le [35] investigated the influence of financial inclusion on carbon emissions by employing the STIRPAT methodology for 31 Asian countries. They recognized that financial inclusion was the reason behind the surge in carbon emissions.

Similarly, Zaidi, Hussain [36] also found a positive impact of financial inclusion on carbon emissions when they utilized the CS-ARDL technique for 23 OECD nations. By employing a similar approach for 5 BRICS nations, Ahmad, Ahmed [37] discovered that financial inclusion was the cause of the surge in carbon emissions. Divergent from the earlier studies, some researchers also found a negative relation between the concerned variables. For instance, the study of Usman, Makhdum [38] revealed a negative linkage between financial inclusion and carbon emissions when they employed AMG tactics to analyze the influence in 5 BRICS nations. Qin, Raheem [39] also found that financial inclusion and cleaner electricity production reduced carbon emissions in E7 nations.

The logical context among financial inclusion, military spending, energy use, and environmental deterioration is represented in Fig 3.

**Fig 3:** Conceptual context of financial inclusion, military, energy use, and environment.

### 2.3. Military spending and environmental sustainability

A few researchers empirically analyzed the nexus between military spending and the environment by taking a panel of countries. Most of these researchers acquired carbon emissions as an indicator to represent the environment. For instance, Khan, Sun [40] analyzed the impact of military on the environment by employing fully modified and updated econometric algorithms for BRICS nations. They discovered that military spending deteriorated environmental quality by enhancing carbon emissions. Moreover, Pata, Destek [41] employed the CS-ARDL technique to investigate the nexus between military and environmental sustainability. They also confirmed that carbon emissions surged due to enhanced military actions in 15 NATO nations.

Unlike other studies, Bradford and Stoner [42] disclosed that the destruction theory was not confirmed for developing nations. Recently, a strong relationship was held between military spending and carbon emissions in rich countries. In addition, Smith and Lengefeld [43] also found similar results while checking the impact of military expenditure on carbon emissions.

On the other hand, the study by Jorgenson, Clark [44] disclosed that militarization had a positive linkage with ecological footprints (indicator for environment) in a panel of 37 nations. Moreover, Bradford and Stoner [12] proved the presence of the theory of destruction in a panel of 142 countries by employing PW and FE panel regression models. They used biological capacity as a measure to represent environmental quality. In a recent study, Qayyum, Anjum [45] documented the positive impact of armed conflicts and military spending on ecological footprints in the South Asian region. Furthermore, Konuk, Kaya [10] concluded that global action is needed to ensure environmental sustainability in place of country-based movements. Still, they presented carbon emissions as a gauge for environmental sustainability, which signifies damage to air quality and cannot cover the definition of environmental sustainability.

### 2.4. Wars (Armed conflicts) and environmental sustainability

Conflicts are a chunk of human civilization, and its history was initiated with the creation of human beings. In addition to physical and psychological suffering, contamination of the environment is also the consequence of wars and conflicts. In this modern era, almost every country around the globe is confronting internal and external conflicts, and our bio-network is degrading due to these conflicts [46]. It is challenging to differentiate war contributors; nowadays, no one can claim that the consequences of war are limited to a specific area as its influences on the environment are not confined to a region or territory [47, 48].

In this modern world, everybody is curious about environmental sustainability. Researchers consider each factor that may influence environmental quality. Still, only a few researchers inspected the association between conflicts and the environment, such as Reuveny, Mihalache-O’Keef [49] found that warfare had harmful impacts on the environment. Still, its influence depended on environmental traits and the type of conflict. It was documented by Pathak [50] that the long-run effects of war on global ecology depended on democracy and income. Hence, high-income nations negatively impact the biological capacity of deprived countries. Furthermore, Ahmed, Ahmad [51] investigated the influence of conflicts and financial risk on environmental sustainability in the Indian context. Their study unveiled that ecological footprints stimulated a reduction in armed conflicts. Apart from these few studies, only Qayyum, Anjum [45] analyzed the combined impact of military spending and armed conflicts on the ecological footprints of South Asia. It was recognized that armed conflicts and military severely affected the environment in both short and long runs.

### 2.5. Terrorism and environmental sustainability

Terrorism is an international phenomenon and nations around the planet spend on military to counter terrorism [52, 53]. In accumulating economic, social, and political influences, terrorism and FDI significantly contribute to carbon emissions [54]. Evidence from India, Turkey, China, and Israel proves that surges in carbon emissions and energy use are caused by terrorism, as terrorist individuals and groups consume massive quantities of energy [55]. Terrorism impacts every aspect of human welfare, including the environment, but this aspect is totally ignored. It was discovered that terrorism deteriorated environmental quality in a panel of some terrorism-affected nations [56]. To achieve environmental sustainability, terrorism should be controlled as it enhanced carbon emissions in the MENA region, while trade and urbanization were negatively related to carbon emissions [21]. Due to the increase in demand and use of high-tech weapons, terrorism has a prominent influence on the environment [57]. Furthermore, terrorism is not only the cause of environmental damage. It also influences the accessibility and supply of drinking water [58].

### 2.6. Institutional quality and environmental sustainability

Recently, various researchers analyzed the influence of institutional quality on ES by taking dissimilar institutional and ES indicators, but the results were ambiguous. For instance, Musa, Jelilov [59] employed a two-step GMM tactic to analyze the impact in the context of 28 EU nations and disclosed that institutional quality was helpful in ES. Moreover, the study of Jahanger, Usman [60] revealed that both IQ and green energy enhanced environmental sustainability when they used FMOLS for a panel of 69 developing nations.

Divergently, Edeme and God [61] & Maji, Saari [62] discovered that IQ had no significant linkage with ES when they employed GMM methodology for a panel of African nations. Dissimilar to all other studies, Riti, Shu [63] utilized press freedom as an indicator for IQ and unveiled that IQ was fruitful for ES. Therefore, this link needs further exaggeration as there are mixed results, and carbon emissions are utilized as an indicator for ES.

### 2.7. Socioeconomic condition and environmental sustainability

In some current studies, researchers attempted to evaluate the association between SEC and ES. Still, most of these studies were conducted by taking a sample of one nation, and the results were also ambiguous. For instance, Zhou, Wang [64] employed the VEC technique for China and divulged that SEC significantly influenced ES. McLean, Bagchi-Sen [65] found that SEC was vital for ES in Peru. Furthermore, Liu, Fujimori [66] determined that SEC had a positive relation with ES, which is more imperative than climatic strategies. In the case of Japan, Shimizu and Kikuchi [67] concluded that ES depended on the execution of socioeconomic driving forces.

On the other hand, Nawaz and Alvi [68] discovered that ES was negatively affected by SEC in Pakistan. In addition, Khan and Hou [69] utilized R&D expenditure as an indicator for SEC, and their results unveiled that ES has deteriorated with betterment in SEC. There is a deficiency of pragmatic literature regarding the relationship between SEC and ES, especially in the panel and global studies case, which creates a massive gap for researchers to investigate this association. The conceptual framework of this study is portrayed in Fig 4.

**Fig 4:** Conceptual framework of the study.

On the basis of theoretical and empirical background, the following hypotheses are constructed for the prime variables of the study.

**H1**: Green energy has a significantly negative impact on ecological footprints.
**H2**: Financial inclusion has a significant and positive influence on ecological footprints.
**H3**: Militarization has a significant positive association with ecological footprints.

## 3. Research methodology and econometric technique

### 3.1 Data and measurement

In this article, an effort has been made to evaluate the influence of green energy, financial inclusion, and military spending on environmental sustainability with global indications. Supplementary factors in this study are war (armed conflicts), terror, institutional quality, and socioeconomic conditions. Panel data composed of 121 nations was collected from dissimilar databases ranging from 2003 to 2022, which was based on the accessibility of the data. Based on the World Bank’s classification, the dataset is divided into 44 high-income, 33 upper-middle-income, and 44 low and lower-middle-income countries.

In this study, ecological footprints (global hectares per capita) represent environmental sustainability, which was suggested by Nathaniel, Yalçiner [70] and Li, Wang [71], while its data has been collected from the Global Footprint Network (GFN). Green energy use is also helpful for environmental sustainability, as employed and suggested by Liu, Alharthi [72], Sharif, Kartal [73], and Sharif, Mehmood [74] which is percentage of total energy consumption and its data is collected from WDI. Furthermore, financial inclusion is another exogenous variable. According to Fareed et al. (2022) & Le et al. (2020), it is a chunk of financial development and plays a vibrant role in poverty reduction. It enables businesses and entities to various financial products and services, including savings, credit, insurance, transactions, and payments. Approachability, quality, and consumption of financial services are termed as financial inclusion. It can impact environmental sustainability because it helps in growing the economy and promotes green investments and technologies. Due to this scenario, PCA of financial inclusion is generated by using certain variables collected through IMF as this database is the best reflector of financial inclusion, and its detail is given in Table 1. Military spending is another explanatory variable and according to the destruction theory, it harms environmental sustainability; its annual data was collected from SIPRI.

**Table 1:** Description of data.

Variable	Symbol	Measurement	H_0_	Source
**a) Dependent Variable**				
Environmental Sustainability	ES	Ecological Footprints (Average GHA per capita)	+/-	GFN
**b) Independent Variables**				
Green Energy	GE	Use of hydropower, solar, wind, geothermal, and biomass energy (% of total energy usage)	-	WDI
Financial Inclusion	FI	PCA index is composed of ATMs/100,000 adults, debit cards/1000 adults, credit cards/1000 adults, commercial bank branches/1000kms, microfinance bank branches/1000kms, credit unions, and credit cooperative branches/1000kms, and financial institutions efficiency (percent)	+	IMF
Military Spending	MS	Military Spending (% of GDP)	+	SIPRI
**(c) Control Factors**				
Armed Conflicts	CON	PCA index including internal and external conflicts (values of these variables ranged from 0–12 in which 0 represented high risk while 12 represented low risk)	+	ICRG
Terrorism	TM	Total number of incidents	+	GTD
Institutional Quality	IQ	PCA index generated from the control of corruption, govt. effectiveness, political stability and absence of violence/terrorism, regulatory quality, rule of law and voice and accountability (% rank)	-	WGI
Socioeconomic Condition	SEC	Socioeconomic Conditions (Conditions ranging from 0–12 in which 0 represents worse condition while 12 represents better condition)	+	ICRG

Besides, armed conflict is PCA generated by the combination of internal and external conflicts as Ahmed, Ahmad [51] and Qayyum, Anjum [45] used these variables, its data is collected from the International Country Risk Guide (ICRG). Global Terrorism Database (GTD) is used to gather data on terrorism, which is comprised of a total number of terrorist incidents per annum as previously utilized by Bildirici and Gokmenoglu [54] & Bildirici [55]. Moreover, institutional quality is represented by the combination of six governance indicators, including control of corruption, govt. effectiveness, political stability and absence of violence/terrorism, regulatory quality, the rule of law, and voice and accountability. The data of these variables is collected from WGI. Socioeconomic condition is the level of riskranging from 0–12 in which 0 represents high risk condition and vice versa, its data was gathered from ICRG. Additionally, missing values were treated by employing Winsor 2 technique. Description of data is provided in Table 1.

### 3.2. Construction of PCA-based indexes

An index signifies an inference of discrete measures by computing a composite measure. Furthermore, the weight index aggregates the products of variable weights and values. For index creation, deciding weights is an imperative stage. PCA is the most appropriate multivariate method Among the other weight-measuring methods [75, 76]. In this study, we utilized different indicators with different units to create indexes, and PCA is the most appropriate technique for constructing such indexes. It is essential to check the suitability of the proxy indicators before converting them into a PCA index. Thus, we utilized Bartlett and Kaiser-Meyer-Olkin (KMO) tests for sphericity and sampling compatibility. Both tests authenticated the appropriateness of the proxy indicators by having significant Chi-square values and KMO values greater than 0.5 [77].

After checking the suitability of the proxy indicators, we constructed PCA indexes in two stages. The initial step comprised identifying less correlated components that resolved the disparity of the proxy indicators. While, the components with higher than one eigenvalue were chosen in the final step.

### 3.3. Empirical model and methodology

The primary aim of this study is to investigate the influence of green energy, financial inclusion, and military policies on environmental sustainability in a sample of 121 nations. The sustainable development theory states that all the environmental, economic, and social goals are interconnected. In comparison, green energy (SDG-7) is a substantial factor in the overall process of sustainable development [78, 79]. It is observed that implementation of all SDGs at local, national, and international levels requires financial inclusivity [80]. In addition, financial inclusion theory emphasizes that access to financial services is the foundation for the overall sustainable development process [81]. On the other side, militarization is momentous for ensuring peace, security, stability, and ocean governance, making it one of the major indicators of SDG-16 [82]. Besides, the treadmill of destruction theory claims that military activities (consuming a major portion of conventional energy) are detrimental to environmental sustainability [83]. We selected prime factors for this study and constructed the following model on these theoretical backgrounds. Moreover, we utilized some control variables related to SDG-16, such as armed conflicts, terrorism, institutional quality, and socioeconomic condition, to generate unbiased outcomes. Following the studies of Ahmed, Ahmad [84] & Gokmenoglu, Taspinar [1], all the variables were converted into log form except PCA-generated variables (financial inclusion, armed conflicts, and institutional quality).


$${ES}_{it}=\gamma_{0}+\gamma_{1}{GEC}_{it}+\gamma_{2}{FI}_{it}+\gamma_{3}{MS}_{it}+\gamma_{4}{CON}_{it}+\gamma_{5}{TM}_{it}+\gamma_{6}{IQ}_{it}+\gamma_{7}{SEC}_{it}+\varepsilon_{it}$$ (1)

In the above equation, i represents a country, t denotes time, *ε*_*it*_ signifies unobserved effects or disturbance error terms, and estimation of unknown parameters is indicated by *γ*_0_, *γ*_1_, *γ*_2_, *γ*_3_, *γ*_4_, *γ*_5_, *γ*_6_ and *γ*_7_. The dynamic model of scrutinizing the influence of military spending, financial inclusion, and green energy on environmental sustainability is given underneath.


$${ES}_{it}=\gamma_{0}+\gamma_{1}{ES}_{it-1}+\gamma_{2}{GEC}_{it}+\gamma_{3}{FI}_{it}+\gamma_{4}{MS}_{it}+\gamma_{5}{CON}_{it}+\gamma_{6}{TM}_{it}+\gamma_{7}{IQ}_{it}+\gamma_{8}{SEC}_{it}+\varphi_{t}+\varepsilon_{it}$$ (2)

In this equation, *ES*_*it*−1_ denotes the time lag value of a dependent variable and *φ*_*t*_ represents the effect of time.

It is mandatory to perform some diagnostic analysis for selecting the prime technique. We started our analysis by checking descriptive statistics. After that, we inspected multicollinearity through a correlation matrix and variance inflation factor (VIF) because issues related to multicollinearity cause biasness and deceptiveness in the outcomes [85]. In panel studies, inspecting cross-sectional dependency is needed because it assists in selecting stationarity tests (first generation for cross-sectionally independent and second generation for cross-sectionally dependent panel) and prime method [86]. Thus, we employed Pesaran and Friedman tests to inspect cross-sectional dependency in the third step. In the next step, we utilized second-generation unit root tests of CIPS and CADF to check the stationarity of the data. In addition, we used the Waterlund and Pedroni co-integration tests to investigate the long-term relationship between study variables.

Finally, the GMM technique is utilized as a prime technique in this empirical investigation because it is suitable for the panel datasets in which the number of cross-sections exceeds the number of time periods (N>T). This study’s dataset comprises 121 nations from 2003–2022 (20 years); therefore, this technique is appropriate for this study. This is an exceptional method to counter specific issues such as cross-sectional dependencies, autocorrelation, measurement of errors, endogeneity biases, and overidentification of constraints [87]. Two-step GMM controls panel heterogeneity. The Wald/Hausman test supports a fixed effect model in three-panel regressions that specifies panel heterogeneity identification. Hence, a dynamic model is evaluated by using system GMM, and two-step sys-GMM is more apposite when the distribution of a dependent variable is not distinguished. The lagged value of environmental sustainability is applied to alter the model into a dynamic one and eradicate autocorrelation in the stationary regression model. Therefore, minimization of the lag effect of the dependent variable (environmental sustainability) will generate reliable results, including long-run anticipating. System GMM not only normalizes autocorrelation, but it also segregates and efficiently examines the outcomes of panel datasets. Hensen-Sargan tests determine the instrument’s reliability and control over-identifying limitations; hence, these tests are operated for comprehensive and premium estimation. The value of Hensen’s test ranges from 0.10 to 0.25, yet it is acceptable up to 0.30. If its value is less than 0.10 or more than 0.30, then the researcher should emphasize it more. The p-value should be less than 0.05 for AR (1) and more than 0.05 for AR (2). The two-step GMM is robust to heteroskedasticity and autocorrelation, making it a more practical technique. Due to these motives, both 2SLS and panel-pooled OSLS are incorporated in this empirical investigation, whereas 2SLS illustrates a specific case of system GMM [88–94].

### 3.4. Inspection of robustness

Primary variables were replaced with alternative variables in system GMM for examining robustness. Reliability of the impact of military spending and other variables on environmental sustainability can be observed by utilizing these methods as a mode to check robustness. The D-K fixed effect standard error tactic and panel quantile regression were employed as substitute methods for supplementary robustness scrutiny. These methods deal with cross-sectional dependence (CD) and integrate heteroskedasticity compatible estimator (HAC), weighted autocorrelation values, and standard errors into weighted HAC values amid residuals and variables. This is endorsed as the most influential method to counter heteroskedasticity, serial and spatial dependence in panel data. In addition to surrounding all kinds of CD and temporal dependence, it also deals with unstable values and panel equilibrium [88, 95]. Fig 5 illustrates the overall methodological procedure followed in this study.

**Fig 5:** Overall methodological procedure.

## 4. Results and discussion

### 4.1. Results of baseline statistics analysis

Descriptive statistics are presented in Table 2, which includes all the info about mean values, amount of observations, standard deviation, and the number of lowest and highest values to better understand the sample and variables. It is observed that all the variables have 2420 observations for 121 countries. Besides, descriptive statistics also summarizes measures of central tendency and gives us an impression of the entire sample through an explanation of data variability. These statistics insinuate that the values of the whole sample are nearer to its mean, which confirms the normal level of dispersal around the mean value. The comprehensive summary and description of these statistics are given in Table 2.

**Table 2:** Descriptive statistics.

Variables	Obs	Mean	Std. Dev.	Min	Max
ES	2420	.978	.731	-.734	2.604
GEC	2420	2.798	1.66	-4.605	4.545
FI	2420	-.055	.471	-.235	3.386
MS	2420	.452	.649	-1.276	2.06
CON	2420	.002	.993	-2.921	1.764
TM	2420	2.281	1.854	-1.099	6.762
IQ	2420	0.000	1.000	-1.602	1.721
SEC	2420	1.597	.568	-.693	2.351

If multiple variables are included in the study, a correlation matrix indicates a higher or lower degree of correlation depending on the obtained values. The amalgamation of the correlation matrix and supplementary statistical practices is utilized to detect multicollinearity problems between the regressors. The correlation matrix of this study has normal values, which show that there is no sign of multicollinearity in the study sample because all the regressor coefficients are below the level of 80%, as suggested by Gujarati [96] and Ullah, Pinglu [88]. The results divulge that all the explanatory variables have a positive association with ES except green energy consumption and terrorism, as shown in Table 3.

**Table 3:** Pairwise correlations.

Variables	ES	GEC	FI	MS	CON	TM	IQ	SEC
ES	1.000							
GEC	-0.524***	1.000						
FI	0.313***	0.113***	1.000					
MS	0.126***	0.118***	0.092***	1.000				
CON	0.257***	-0.317***	-0.021	0.110***	1.000			
TM	-0.242***	0.239***	-0.078***	-0.054**	-0.297***	1.000		
IQ	0.533***	-0.012	0.344***	-0.235***	0.379***	-0.260***	1.000	
SEC	0.631***	0.144***	0.309***	-0.373***	0.323***	-0.230***	0.516***	1.000

*** p<0.01 (1%)

** p<0.05 (5%)

* p<0.1 (10%)

Furthermore, the variance inflation factor (VIF) was also employed in the study for additional authorization about multicollinearity issues in the sample. Several studies show that the VIF value should not exceed 5 [85]. As shown in Table 4, all the VIF values meet the recommended criteria by confirming no multicollinearity issue in the study sample.

**Table 4:** Variance inflation factor with time effect.

Variables	VIF with Time effect (1–2)		VIF without Time effect (1–2)	
	VIF	1/VIF	VIF	1/VIF
GEC	1.378	.726	1.373	.728
FI	1.291	.774	1.283	.779
MS	1.532	.653	1.521	.658
CON	1.546	.647	1.535	.651
TM	1.227	.815	1.172	.853
IQ	2.406	.416	2.402	.416
SEC	2.384	.42	2.373	.421
2004. year	1.986	.503		
2005. year	1.977	.506		
2006. year	2.002	.499		
2007. year	2.092	.478		
2008. year	2.014	.497		
2009. year	1.99	.503		
2010. year	2.053	.487		
2011. year	2.008	.498		
2012. year	2.112	.474		
2013. year	2.099	.477		
2014. year	2.14	.467		
2015. year	2.256	.443		
2016. year	2.146	.466		
2017. year	2.147	.466		
2018. year	2.131	.469		
2019. year	2.095	.477		
2020. year	2.117	.472		
2021. year	2.178	.459		
2022. year	2.109	.462		
**Mean VIF**	**1.972**	.	**1.666**	.

### 4.2. Results of cross-sectional dependency

In this era of globalization, economies are cohesive, which enhances the chance of dependency in the cross-sections. Consequently, a shock can be easily transferred from one nation to another, and correlation between cross-sections augments. Therefore, it is mandatory to test cross-sectional dependency issues to generate unbiased outcomes due to size misrepresentations, stationarity, and cointegration. The current study uses the Pesaran panel cross-sectional dependence test because it is specially developed for the panels having larger cross-sections than time [86, 97]. In addition, Friedman’s test is also employed for further authentication. It is found that the p-values of both tests are significant at a one percent level of significance by rejecting the null hypothesis of cross-sectional independence, as shown in Table 5.

**Table 5:** Results of cross-sectional dependence tests.

Test	Random effect	Fixed effect
Pesaran	16.557***	15.670***
Friedman	10.810***	10.902***

*** p<0.01 (1%)

** p<0.05 (5%)

* p<0.1 (10%)

### 4.3. Second-generation unit root test

Based on the outcomes of cross-sectional dependence, the generation of the unit-root test is decided. If the panel is cross-sectionally independent, it is better to utilize first generation unit root tests. Second-generation unit root tests are most feasible if the panel is cross-sectionally dependent [98]. As the panel is cross-sectionally dependent, thus, CIPS and CADF second-generation unit tests have been utilized for the dataset. It is divulged that ES, CON, TM, IQ, and SEC are stationary at a level. At the same time, GEC, FI, and MS are stationary at the first difference in the CIPS unit root test, as shown in Table 6. FI, CON, and IQ are stationary at a level, while other variables are stationary at the first difference in the CADF unit root test. On the basis of these results, the null hypothesis is rejected and the alternative hypothesis is accepted, which validates that all the variables included in the study are stationary at the level or first difference. Besides, these results also favor the fitness of the proposed model and the advancement of the outcomes.

**Table 6:** Results of second-generation unit root tests.

	CIPS			CADF		
Variables	At Level	First Difference	I(d)	At Level	First Difference	I(d)
ES	-2.605**	-	I(0)	-1.906	-2.547***	I(1)
GEC	-2.257	-4.454***	I(1)	2.155	-2.391***	I(1)
FI	-2.051	-3.099***	I(1)	-2.126***	-	I(0)
MS	-2.451	-4.130***	I(1)	1.796	-2.530***	I(1)
CON	-2.757***	-	I(0)	-2.404***	-	I(0)
TM	-3.514***	-	I(0)	-0.487	-5.201***	I(1)
IQ	-2.938***	-	I(0)	-2.418*	-	I(0)
SEC	-2.549*	-3.417***	I(1)	-0.960	-2.970***	I(1)

*** p<0.01 (1%)

** p<0.05 (5%)

* p<0.1 (10%)

### 4.4. Cointegration tests

Westerlund test (2007) and Padroni test (2004) are employed for this particular study to investigate the panel model’s cointegration. Both of these tests validate that the panel is cointegrated, as depicted in Table 7. The Westerlund test is the most advanced and modern practice to investigate cointegration in panel datasets. By rejecting the null hypothesis, results reveal that panels are cointegrated at a 1% significance level with a value of -6.9321, and the detail of these results is depicted in Table 7.

**Table 7:** Tests for the cointegration.

Detail	Value		Accepted/Rejected
**Westerlund test for cointegration**			
Variance ratio	-6.9321 ***		Ha: All panels are cointegrated (Accepted)
Number of panels: 121			
Avg. number of periods: 19.85			
Cointegrating vector: Panel specific			
Panel means: Included			
Time trend: Included			
AR parameter: Same			
Cross-sectional means removed			
**Pedroni test for cointegration**			
Modified Phillips-Perron t	4.3417***		Ha: All panels are cointegrated (Accepted)
Phillips-Perron t	-23.0661***		
Augmented Dickey-Fuller t	-21.0659***		
Number of panels = 121		Cointegrating vector: Panel specific		
Panel means: Included		Kernel: Bartlett		
Avg. number of periods = 18.85		Time trend: Included		
Augmented lags: 1		Lags: 2.00 (Newey-West)		
Cross-sectional means removed		AR parameter: Panel specific		

Standard errors in parentheses

*** p<0.01 (1%)

** p<0.05 (5%)

* p<0.1 (10%)

### 4.5. Dynamic impact of green energy, financial inclusion, and military on ecological footprints

If the panel is cross-sectionally dependent, then the Augmented mean group (AMG), mean group (MG), and pooled mean group (PMG) can produce deceptive outcomes. In large and cross-sectionally dependent panels, the generalized method of moments (GMM) is the most suitable pragmatic technique [99, 100]. Therefore, we selected a two-step system GMM technique for this study. This section presents outcomes related to environmental sustainability with the assistance of the two-step system GMM. Furthermore, the results of the robustness check (by using substitute variables and techniques, including D-K regression) are also demonstrated in Table 8. The final model is a two-step system GMM, and it is designated based on its criteria and Wald test outcomes. The results of this final model are portrayed in the first column, and it is disclosed that the lag value of a dependent variable (ES) is 0.495 at a 1% significance level. This value specifies that ES will be influenced by 0.495% with a 1% variation in exogenous variables. Moreover, green energy consumption benefits environmental sustainability. It is witnessed from the outcomes that a 1% surge in the consumption of GEC will significantly reduce ECFTs by 5.9%.

**Table 8:** Results of green energy, financial inclusion, and military dynamic factors affecting environmental sustainability on a global level.

Dep. Variable	(1)	(2)	(3)	(4)
	Two-step Sys-GMM (1–3)			D-K F.E. Regression
	E. S Main Model	E. S Robust Model	E.S Robust Model	E. S Robust Model
Environmental Sustainability (t-1)	0.495***	0.496***	0.475***	
	(0.032)	(0.032)	(0.026)	
Green Energy	-0.059*** (0.017)	-0.059*** (0.017)	-0.064*** (0.014)	-0.170*** (0.016)
Financial Inclusion	0.070***	0.063***	0.054***	0.126** (0.032)
	(0.023)	(0.024)	(0.021)	
Military Spending	0.069*** (0.023)	0.069*** (0.023)	0.040* (0.023)	0.027* (0.015)
Terrorism	0.014**	0.014**	0.008*	0.008**
	(0.006)	(0.006)	(0.005)	(0.003)
Institutional Quality	0.143***	0.144***	0.111***	0.078*
	(0.018)	(0.018)	(0.017)	(0.027)
Socioeconomic Conditions	0.163***	0.164***	0.173***	0.078*
	(0.034)	(0.034)	(0.029)	(0.027)
Conflicts	0.023*		0.019*	0.019***
	(0.012)		(0.011)	(0.004)
External Conflicts (Robust)		0.146*		
		(0.085)		
	(0.034)	(0.034)	(0.029)	(0.027)
Health Expenditure (Robust)			0.160***	
			(0.023)	
i.Year Effect	YES	YES	YES	YES
Observations	2,299	2,299	2,299	2,299
**Diagnostic Analysis**				
AR1	-1.532	-1.537	-1.540	
AR1 p-value	0.016	0.014	0.022	
AR2	1.546	1.559	1.663	
AR2 p-value	0.122	0.119	0.0964	
Sargan	150.1	149.4	126.5	
Hansen	58.06	57.79	62.93	
Hansen p-value	0.203	0.210	0.190	
Chi2/Wald test	18984	19487	22351	
Chi2 p-value	0	0	0	
J-stat, Instruments	76	76	81	
within R-squared				0.6867
Prob > F				0.0000
No. of Countries	121	121	121	121

Standard errors in parentheses

*** p<0.01 (1%)

** p<0.05 (5%)

* p<0.1 (10%)

Note: We took the log of ES, GE, MS, TM & SEC

Furthermore, a composite of financial inclusion also has a positive and significant association with ecological footprints at a 1% level. As indicated by its value of 0.070, a 1% positive change in financial inclusion will cause a 7% increase in ecological footprints (7% harmful to environmental sustainability) because an enhancement in financial inclusion promotes an increase in the number of buildings, equipment, ATMs, staff and visitors as well, which are the causes for environmental deterioration. In addition, the coefficient of military spending is positive (0.069) at the significance level of 1%, which divulges that a 1% increase in military expenditure will enhance ecological footprints by 6.9%. It means a surge in military spending harms environmental sustainability, proving the prevalence of the theory of destruction globally.

By sanctioning all the theoretic validations, the outcomes of this study reveal that a 1% upsurge in a composite of armed conflicts causes 2.3% harm to ES (by increasing ECFTs) at a 10% significance level. Likewise, the outcomes of this particular study revealed that ECFTs would be significantly enhanced by 1.4%, with a 1% upsurge in terrorist incidents at a 5% significance level.

Composite of Institutional quality has a significant positive linkage with ECFTs, and it is discovered that ECFTs will increase (ES will be harmed) by 14.3% with a 1% increase in IQ. They argue that serious developments are required in IQ because the promotion of investing in the public and private green energy sector is dependent on it. Additionally, a 1% positive change in socioeconomic conditions will cause a 16.3% increase in ECFTs by deteriorating ES. There are several reasons behind it, such as urbanization, population, economic activity, and city progress due to the surge in SEC, which are considered significant factors in deteriorating ES.

In addition, several diagnostic tests are performed to endorse outcomes further and guarantee precise inference. The results of these diagnostic tests are depicted in the first column of Table 8. It is divulged that the employed model has no serial and auto-correlation because the p-value of AR (1) is less than 5%. Furthermore, a p-value of AR (2) is more than 5%, which is an indication of the appropriateness of the system GMM technique for the current sample (N = 121>T = 20). Moreover, the Wald/chi-square test and F-statistics have significant p-values at the 1% level, symbolizing the suitability of the applied model. The statistic values of the Hansen and Sargan tests are 58.06 and 150.1, correspondingly, and the p-value of the Hansen test is 0.203; consequently, these tests corroborate the reliability of instruments and restrictions of over-identifying by accepting the null hypothesis. Henceforth, the outcomes of all the methodical tests fulfil standards and assumptions, which effectively demonstrates the consistency and accuracy of the applied procedure.

Furthermore, Table 9 demonstrates the dynamic nexus of green energy, financial inclusion, military spending, and ecological footprints in different income level groups of countries using the two-step system GMM technique. Based on World Bank classifications, countries are divided into three income level groups: high-income, upper-middle income, and low and lower-middle-income countries. The outcomes endorse the dynamic nature of nexus in all income level groups. It is discovered that a one % surge in green energy usage significantly reduces ecological footprints in high-income, upper-middle-income, and low and lower-middle-income countries by 3.3, 1.3, and 2.8%, respectively. Moreover, financial inclusion greatly enhances ecological footprints by 10.6 and 21.7 in high-income and upper-middle-income countries, respectively. Still, it has a negative and non-significant impact on ecological footprints in low and lower-middle-income countries. Moreover, a one % increase in militarization significantly augments ecological footprints by 34.7% and 4.7% in high-income and low- and lower-middle-income countries, respectively. Still, in upper-middle-income countries, ecological footprints are significantly reduced by 13%.

**Table 9:** Results of green energy, financial inclusion, and military dynamic factors affecting environmental sustainability on different income level groups.

	(1)	(2)	(3)
Dep. variable	High income	Upper-middle income	Low and lower-middle income
Ecological footprints (t-1)	0.513***	0.536***	0.447***
	(0.078)	(0.204)	(0.035)
Green energy	-0.033***	-0.013**	-0.028***
	(0.009)	(0.018)	(0.002)
Financial inclusion	0.106*	0.217**	-0.019
	(0.088)	(0.141)	(0.115)
Military expenditure	0.347**	-0.130*	0.047***
	(0.138)	(0.075)	(0.013)
Armed conflicts	-0.111	0.047***	0.081**
	(0.077)	(0.110)	(0.041)
Terrorism	-0.009***	0.012*	0.025**
	(0.002)	(0.050)	(0.032)
Institutional quality	0.442***	-0.037**	-0.011***
	(0.140)	(0.108)	(0.060)
Socioeconomic condition	0.115*	0.042***	0.321***
	(0.060)	(0.086)	(0.037)
i. year effect	yes	yes	yes
Observations	836	627	836
Number of countries	44	33	44
AR1	-3.141	-2.152	-1.028
AR1 p-value	0.00169	0.0314	0.0204
AR2	1.375	1.083	0.977
AR2 p-value	0.169	0.279	0.329
Sargan	75.71	40.58	128.4
Sargan p-value	8.13238	7.00925	5.34529
Hansen	20.09	7.392	18.74
Hansen p-value	0.577	0.998	0.661
J-stat	29	17	32
Chi2	30516	44193	33783
Chi2 p-value	0	0	0

Standard errors in parentheses

*** p<0.01

** p<0.05

* p<0.1

Additionally, armed conflicts and terrorism have a significant and positive association with ecological footprints in upper-middle and low and lower-middle-income countries. In contrast, in high-income nations, armed conflicts and terrorism have a non-significant and significantly negative relation with ecological footprints, respectively. Moreover, betterment in institutions reduces ecological footprints in upper-middle and low and lower-middle-income countries, but a significant and positive link is found in high-income nations. Improving socioeconomic conditions is detrimental to environmental sustainability because it positively relates to ecological footprints in all income level groups. Similar to post-analysis outcomes of global level data, the results of post-diagnostic tests of sub-divided income level groups also endorse the reliability of applied methods and outcomes.

### 4.6. Outcomes of time effect

Outcomes rendering time influence are depicted in Table 10. It is discovered that positive changes in ECFTs have occurred during all the study periods except 2004, 2005, and 2008. It means the environment has significantly deteriorated in all this study period except in 2004, 2005, and 2008. Moreover, insignificantly positive changes in ECFTs were witnessed in 2004 and 2005, which became significant in the second robust model and DK regression at 1% significance. On the other hand, negative but insignificant influences on ECFTs were discovered in 2008, possibly due to the global economic crisis of 2008.

**Table 10:** Results of time effect through two-step system GMM and D-K regression.

	(1)	(2)	(3)	(4)
	Two-step system GMM (1–3)			D-K regression
Dep. Variable	E. S Main Model	E. S Robust Model	E.S Robust Model	E. S Robust Model
Base year (2003)				
2004bn. year	0.012	0.013	0.036***	0.028***
	(0.012)	(0.012)	(0.011)	(0.002)
2005	0.016	0.017	0.038***	0.034***
	(0.013)	(0.013)	(0.012)	(0.002)
2006	0.033***	0.034***	0.058***	0.047***
	(0.011)	(0.011)	(0.010)	(0.003)
2007	0.047***	0.048***	0.070***	0.058***
	(0.011)	(0.011)	(0.010)	(0.003)
2008	-0.002	-0.001	0.011	0.027***
	(0.012)	(0.012)	(0.011)	(0.002)
2009	0.053***	0.054***	0.070***	0.058***
	(0.010)	(0.010)	(0.009)	(0.003)
2010	0.042***	0.043***	0.060***	0.062***
	(0.010)	(0.010)	(0.009)	(0.003)
2011	0.022**	0.023**	0.040***	0.044***
	(0.009)	(0.009)	(0.008)	(0.004)
2012	0.041***	0.042***	0.056***	0.061***
	(0.009)	(0.009)	(0.008)	(0.008)
2013	0.018***	0.018***	0.022***	0.018***
	(0.007)	(0.007)	(0.006)	(0.005)
2014	0.030***	0.030***	0.038***	0.027***
	(0.006)	(0.006)	(0.006)	(0.005)
2015	0.032***	0.033***	0.034***	-0.013
	(0.005)	(0.005)	(0.005)	(0.010)
2016	0.035***	0.035***	0.041***	0.027***
	(0.004)	(0.004)	(0.004)	(0.006)
2017	0.030***	0.030***	0.035***	0.033***
	(0.006)	(0.006)	(0.006)	(0.006)
2018	0.028***	0.028***	0.035***	0.029***
	(0.005)	(0.005)	(0.006)	(0.005)
2019	0.034***	0.034***	0.039***	0.030***
	(0.006)	(0.006)	(0.005)	(0.005)
2020	0.037***	0.037***	0.041***	0.030***
	(0.006)	(0.006)	(0.005)	(0.005)
2021	0.035***	0.035***	0.040***	0.031***
	(0.006)	(0.006)	(0.005)	(0.005)
2022	0.032***	0.032***	0.039***	0.031***
	(0.005)	(0.005)	(0.005)	(0.005)

Standard errors in parentheses

*** p<0.01 (1%)

** p<0.05 (5%)

* p<0.1 (10%)

### 4.7. Outcomes of robustness

The principal model’s cogency and outcomes are authorized using triple robustness, as represented in columns (2, 3 & 4) of Table 8. Initially, external conflicts are replaced with a variable of armed conflicts. Then, health expenditure is added with the rest of the primary variables to inspect the validity of outcomes by using the two-step system GMM technique. The results of all the analytical tests and principal methods are demonstrated in columns 2 and 3, which specify that all the assumption criteria are fulfilled. In accumulation to authenticating model steadiness and reliability in robustness, retrieved outcomes also guarantee accuracy in inferences and overall fitness of the pragmatic model. Like a composite of armed conflicts, external conflicts also have a significant and positive impact on ECFTs (detrimental for ES), with a change of 14.6% at a 10% significance level. Moreover, a 1% positive change in health expenditure will cause a 16% enhancement in ECFTs at a 1% significance level.

Including these substitute variables in robust models has not changed overall outcomes related to the primary variables, as seen in Columns 2 & 3 of Table 8. Henceforth, the findings of the first two robust models strongly authorize the cogency of the pragmatic model. Furthermore, diagnostic tests validate the results by certifying correctness in inference and fulfilling specific criteria. These findings are detailed in second and third columns of Table 8.

After inspecting robustness by replacing variables, an alternative method (D-K fixed effect regression) is used to finalize all the robustness processes. This method specifies that there are no endogeneity issues and cross-sectional dependence in the outcomes, which approves the reliability of the two-step system GMM. These findings are described in the 4^th^ column of Table 8.

In addition, the robustness of the outcomes of income level groups is checked by applying two alternative techniques, including quantile and Driscoll-Kraay regressions. The results of these techniques are demonstrated in Table 11.

**Table 11:** Outcomes of the robustness through quantile and D-K regressions in different income level groups.

	(1)	(2)	(3)
Dep. variable	High income	Upper-middle income	Low and lower-middle income
	(Quantile regression)	(D-K regression)	(Quantile regression)
Green energy	-0.032***	-0.024***	-0.008***
	(0.008)	(0.003)	(0.001)
Financial inclusion	0.153*	0.147***	-0.036
	(0.108)	(0.021)	(0.101)
Military expenditure	0.395***	-0.046*	0.010***
	(0.084)	(0.038)	(0.022)
Armed conflicts	-0.051	0.011*	0.030*
	(0.146)	(0.032)	(0.032)
Terrorism	-0.014***	0.019**	0.001***
	(0.005)	(0.032)	(0.008)
Institutional quality	1.051***	-0.020***	-0.103*
	(0.188)	(0.031)	(0.053)
Socioeconomic condition	0.420***	0.081***	0.090***
	(0.097)	(0.025)	(0.023)
i. year effect	yes	yes	yes
Observations	880	660	880
Number of countries	44	33	44
Pseudo R-squared	0.262		0.340
R-squared		0.5913	
Prob>F		0.0000	

Standard errors in parentheses

*** p<0.01

** p<0.05

* p<0.1

The robust models also produced similar outcomes to the prime model, which authenticates all the results regarding income level groups. Moreover, the value of Pseudo R-square in quantile regression and the values of R-square and F-statistic in D-K regression further corroborate the consistency of the pragmatic procedure.

### 4.8. Discussion of key findings

This study empirically scrutinizes and deliberates the influence of green energy, financial inclusion, militarization, and other supplementary variables on environmental sustainability by taking a sample of 121 nations from 2003 to 2022. For a global and sub-group level comparison, the dataset is divided into three income-level groups comprised of 44 high-income, 33 upper-middle-income, and 44 low and lower-middle-income countries. While analyzing the nexus, it is found that consumption of green energy is negatively linked with ecological footprints at all global and income group levels, which is aligned with Adekoya, Ajayi [30] and Mujtaba, Jena [101]. By accepting the proposed hypothesis, these outcomes also validate the foundations of sustainable development theory and COP-28. Because green energy sources contribute minimum to greenhouse gases and utilize fewer resources than conventional energy sources, further developments in technology and sustainability practices are likely to nullify the footprints of green energy sources.

In contrast, financial inclusion has a positive influence on ecological footprints worldwide, high income, and upper-middle income levels, as proposed in the hypothesis and found by Fareed, Rehman [26] and Singh, Raza [102], but a non-significant relation is discovered in low and lower-middle income countries. It is argued by Jingpeng, Ullah [103] that financial inclusion boosts economic and business activities, which are the major causes of environmental damage. People from low-income countries face severe economic and survival pressure with limited access to green energy technologies and limited capacity to recover from economic shocks, making them more vulnerable to environmental sustainability.

Furthermore, military spending was also found to be detrimental to environmental sustainability by positively associating with ecological footprints at all group levels except upper-middle-income countries. These outcomes are consistent with Chang, Chen [104] and Eregha, Vo [105] findings. However, militarization is beneficial for environmental sustainability for upper-middle-income countries because it has a negative linkage with ecological footprints, as Zhu et al. (2023) found. The findings reveal that the theory of the treadmill of destruction holds for all categories except upper-middle-income countries. Wide usage of fossil fuels and natural resources, training, and weapon testing make the military detrimental to environmental sustainability in all the major categories. However, military spending in non-battle activities can be beneficial for environmental sustainability.

Moreover, armed conflicts and terrorism negatively affected environmental sustainability by having a positive linkage with ecological footprints at global, upper-middle income, and low and lower-middle income levels as of the outcomes of Qayyum, Anjum [45], Bildirici [55], and Tahir, Burki [21]. Divergently, armed conflicts are non-significant, and terrorism negatively affects ecological footprints in high-income countries. The economies of high-income countries are based on trade, investments, industrialization, manufacturing, and socioeconomic activities coupled with massive urbanization. While the surge in terrorist incidents directly influences these activities in high-income countries, which are the major causes of environmental deterioration [106].

Moreover, socioeconomic condition also has a significant and positive relation with ecological footprints at all levels; however, institutional quality significantly enhances ecological footprints at a global and high-income level, which is parallel to the outcomes of Abid, Marchesani [107], Maji, Saari [62], Khan and Hou [69] & Nawaz and Alvi [68]. Whereas institutional quality significantly reduces ecological footprints in upper-middle-income and low and lower-middle-income countries, these outcomes are consistent with the studies of Ahmad, Ahmed [108] and Jahanger, Usman [60].

Furthermore, the outcomes of the VIF test disclose that multicollinearity has not influenced overall results. The findings of the second-generation unit root test divulge that all the data is stationary at level or first difference, which corroborates the fitness of the dynamic nature of data. In addition, cointegration tests (Westerlund & Pedroni) prove that all the panels are cointegrated by refusing the null hypothesis. Collectively, these diagnostic tests recommend the application of comprehensive valuation techniques to get systematic answers.

The current study applies the two-step system GMM method after confirming the reliability and fulfilment of basic criteria by various analytic tactics such as AR1, AR2, Sargan test, Hansen test, Wald test, and J-statistics. Besides, the outcomes of this method are further verified by employing alternative variables (external conflicts and health expenditure) and substitute techniques (Quantile and D-K regression). The findings of the principal model reveal that green energy use is significantly beneficial for ES at all global and income levels. At the same time, financial inclusion, military spending, armed conflicts, institutional quality, and socioeconomic conditions have a significant destructive influence on ES at global and most income level groups. Dissimilarly, financial inclusion, and armed conflicts have a non-significant impact on ES in low-income and high-income countries. In addition, institutional quality enhances ES in upper-middle and low and lower-middle-income countries, while terrorism enhances ES in high-income countries.

While inspecting robustness, it is found that alternative variables comprising external conflicts and health expenditure also significantly deteriorate ES without changing the findings of the principal model. Finally, the Quantile and D-K regression outcomes also support the reliability of the two-step GMM model by confirming the absence of endogeneity and cross-sectional dependency issues.

## 5. Conclusion and policy implications

In this study, efforts have been made to analyze the impact of green energy use, financial inclusion, military, armed conflicts, terror, institutional quality, and socioeconomic conditions on environmental sustainability in 121 nations from 2003 to 2022. The dataset is divided into 44 high-income, 33 upper-middle-income, and 44 low and lower-middle-income countries for better contribution to existing literature. The dependent variable ES is based on ecological footprints, while green energy consumption, financial inclusion, and military spending are independent variables. Besides, other determinants comprised of armed conflicts, terrorism, institutional quality, and socioeconomic conditions are included as control variables. The outcomes revealed that there is no issue of multicollinearity in the dataset, and the panel is cross-sectionally dependent.

Furthermore, the results of the unit root (CIPS and CADF) and cointegration tests (Westerlund & Pedroni tests) divulge that data is stationary at the level and the panel is cointegrated correspondingly. Moreover, the association between explained variables and environmental sustainability is evaluated with a two-step system GMM, and the results’ robustness is further inspected using alternative variables and methodologies, including panel Quantile and Driscoll-Kraay (D-K) regressions. It is found that green energy use benefits ES because of their negative and significant linkage with ECFTs at all levels.

On the other hand, military spending, financial inclusion, armed conflicts, terrorism, institutional quality, and socioeconomic conditions are detrimental to ES because these variables positively affect ECFTs at global and most of the income level groups. Dissimilarly, financial inclusion and armed conflicts have a non-significant influence on ecological footprints in low-income and high-income countries, respectively. Furthermore, institutional quality enhances ES in upper-middle and low and lower-middle-income countries by negatively affecting ecological footprints. At the same time, terrorism significantly reduces ecological footprints in high-income countries.

Based on outcomes, it is suggested that governments and policy designers should promote the adoption of green energy by providing regulatory support such as relief in taxes, tariffs, and green energy standards. Furthermore, policymakers should set environmental targets, and government bodies should ensure the implementation of these policies to achieve recent climatic goals such as COP-28. Assuming the latest global attention for sustainability, a viable ground should be provided for green energy investors because investing in green energy projects yields long-term returns. Fossil fuel prices are unstable due to the volatility of energy markets. Energy companies can benefit from green energy sources, which can assist in accomplishing climatic goals by stabilizing energy prices. Governments and stakeholders should encourage businesses and corporations to adopt green energy technologies, which are more cost-efficient than conventional energy.

Moreover, public and private organizations should cooperate to launch community-based green energy projects. These projects can also enhance employment and green innovation in local communities. Conversely, environmental organizations should collaborate with stakeholders to provide general awareness about the environment and green energy transition.

Although financial inclusion develops the economy, all the growing economies should allocate specific portions of their resources for environmental conservation. Moreover, government and private institutions should design policies that encourage financially included businesses and entities to invest in green technologies and products. The financial sector should take substantial initiatives to digitalize the financial system because it can lower environmental damage by reducing finance-related energy consumption activities and reliance on paper money (the primary cause of deforestation). In addition, the financial sector should collaborate with other public and private organizations to provide finance for green community initiatives and financial products such as climate insurance, green bonds, and green energy installations.

Besides, government agencies and military officials should introduce particular environmental standards and regulations within the military to lessen environmental deterioration. Environmental organizations can play their role by negotiating with military officials to encourage sustainable practices in military operations. Furthermore, policymakers should design policies to promote green energy use in the military sector to reduce environmental damage. Weapons manufacturers should use green technologies to ensure sustainable manufacturing procedures, and they should also have a dialogue with governments for responsible utilization of military weapons. Moreover, local environmental and media activists can put a pressure on the government to ensure sustainable practices during military activities by providing environmental awareness to the general public. Military expenditure is divided into two major categories: battle and non-battle. Instead of spending on the battle, authorities should prefer non-battle defense spending because spending on battle ammo entails non-green energy consumption. Governments, organizations, and concerned authorities should take substantial initiatives to promote peace at national and international levels by resolving armed conflicts and overcoming terrorism incidents to sustain the environment. Education and awareness about terrorism should be given to individuals and entities on each level so they do not engage in terrorist activity. Additionally, political victimization, religious extremism, and economic conditions are some basic reasons for people’s involvement in terrorist activities. Joint action is required to take substantial steps to deal with these issues.

Institutional quality requires further improvements at a global level, especially in high-income countries, because it also jeopardizes global environmental sustainability. There is a need for sturdy and inclusive institutions that should have a prominent capability to encourage green energy consumption by reducing conventional energy use. Institutions should also endorse private sector investments in green energy. Individuals, economic entities, investors, financial institutions, and social organizations feel frightened due to terrorism, which hinders overall social and economic activity in high-income countries. These actions require a massive amount of conventional energy, the fundamental cause of environmental damage. Education and awareness about environmental sustainability should be given to individuals and entities on each level so that they can concentrate more on the ecological damage caused by their daily activities.

The outcomes of this study reveal that improving socioeconomic conditions hampers environmental sustainability worldwide. A surge in urbanization, population, infrastructure, and other economic actions is the chief cause of environmental damage on a global level. Governments and institutions should have absolute control over these factors by implementing environmental laws. Besides, authorities should discourage deforestation caused by these socioeconomic factors and promote plantation and green energy consumption.

This study is limited to 121 nations to estimate the dynamic influence of green energy, financial inclusion, military, armed conflicts, terror, institutional quality, and socioeconomic conditions on environmental sustainability. The dataset of these variables ranges from 2003–2022 because data on financial inclusion indicators is available within this range. Therefore, this is the best possible dataset based on accessibility of time range and number of nations.

In the future, researchers can contribute further by including other socioeconomic factors linked with green energy transition in studying the nexus between green energy and environmental sustainability. Furthermore, digital financing, technically advanced institutions, green innovations, and green funding can also play a vital role in the transition to green energy; hence, these factors can also be included in environment-related studies. Moreover, this nexus can also be analyzed and compared by employing dissimilar methodologies and regions.

## Supporting information

S1 Dataset (XLSX)

## References

[1] GokmenogluK.K., TaspinarN., and RahmanM.M., Military expenditure, financial development and environmental degradation in Turkey: a comparison of CO2 emissions and ecological footprint. International Journal of Finance & Economics, 2021. 26(1): p. 986–997.

[2] KirikkaleliD. and AdebayoT.S., Do renewable energy consumption and financial development matter for environmental sustainability? New global evidence. Sustainable Development, 2021. 29(4): p. 583–594.

[3] AdebayoT.S., et al., Endorsing sustainable development in BRICS: The role of technological innovation, renewable energy consumption, and natural resources in limiting carbon emission. Science of the Total Environment, 2023. 859: p. 160181. doi: 10.1016/j.scitotenv.2022.160181 36384177

[4] KartalM.T., et al., Do nuclear energy and renewable energy surge environmental quality in the United States? New insights from novel bootstrap Fourier Granger causality in quantiles approach. Progress in Nuclear Energy, 2023. 155: p. 104509.

[5] SunY., et al., Renewable energy transition and environmental sustainability through economic complexity in BRICS countries: Fresh insights from novel Method of Moments Quantile regression. Renewable Energy, 2022. 184: p. 1165–1176.

[6] MukalayiN.M. and Inglesi-LotzR., Digital financial inclusion and energy and environment: Global positioning of Sub-Saharan African countries. Renewable and Sustainable Energy Reviews, 2023. 173: p. 113069.

[7] MurshedM., et al., The impacts of renewable energy, financial inclusivity, globalization, economic growth, and urbanization on carbon productivity: Evidence from net moderation and mediation effects of energy efficiency gains. Renewable Energy, 2022. 196: p. 824–838.

[8] OzturkI. and UllahS., Does digital financial inclusion matter for economic growth and environmental sustainability in OBRI economies? An empirical analysis. Resources, Conservation and Recycling, 2022. 185: p. 106489.

[9] BiscioneA. and CarusoR., Military expenditures and income inequality evidence from a panel of transition countries (1990–2015). Defence and Peace Economics, 2021. 32(1): p. 46–67.

[10] KonukF., et al., The relationship between military expenditures, financial development and environmental pollution in G7 Countries. Journal of the Knowledge Economy, 2023: p. 1–16.

[11] BargaouiS.A. and NouriF.Z., Dynamic panel data analysis of CO2 emissions driving forces. Journal of Economics Studies and Research, 2017. 2017(2017): p. 1–18.

[12] BradfordJ.H. and StonerA.M., IN COMPARATIVE PERSPECTIVE: A PANEL STUDY OF THE BIOLOGICAL CAPACITY OF NATIONS, 1961–2007. 2014.

[13] GaoS., et al., Financial inclusion empowering sustainable technologies: Insights into the E-7 economies from COP28 perspectives. Technological Forecasting and Social Change, 2024. 201: p. 123177.

[14] ZhuW., et al., How military spending, economic growth, and renewable energy impacts ecological footprints in Next Eleven nations. Environmental Science and Pollution Research, 2023: p. 1–11.10.1007/s11356-023-29633-z37697190

[15] StrezovV., EvansA., and EvansT.J., Assessment of the economic, social and environmental dimensions of the indicators for sustainable development. Sustainable development, 2017. 25(3): p. 242–253.

[16] CuiL., et al., Exploring the role of renewable energy, urbanization and structural change for environmental sustainability: Comparative analysis for practical implications. Renewable Energy, 2022. 184: p. 215–224.

[17] O’ReillyG., Achieving a Sustainable Future: The Geographical Centrality of UN SDG-16, Peace, Justice and Strong Institutions, in Sustainable Development Goals in Europe: A Geographical Approach. 2023, Springer. p. 329–349.

[18] AshaP., et al., Role of machine learning in attaining environmental sustainability. Energy Reports, 2022. 8: p. 863–871.

[19] TóthováD. and HeglasováM., Measuring the environmental sustainability of 2030 Agenda implementation in EU countries: How do different assessment methods affect results? Journal of Environmental Management, 2022. 322: p. 116152.

[20] AbidN., et al., Financial development and green innovation, the ultimate solutions to an environmentally sustainable society: evidence from leading economies. Journal of Cleaner Production, 2022. 369: p. 133223.

[21] TahirM., BurkiU., and AzidT., Terrorism and environmental sustainability: Empirical evidence from the MENA region. Resources, Environment and Sustainability, 2022. 8: p. 100056.

[22] PereiraP., et al., The Russian-Ukrainian armed conflict impact will push back the sustainable development goals. 2022, Elsevier.

[23] UsmanO., AlolaA.A., and Saint AkadiriS., Effects of domestic material consumption, renewable energy, and financial development on environmental sustainability in the EU-28: Evidence from a GMM panel-VAR. Renewable Energy, 2022. 184: p. 239–251.

[24] XuB. and XuR., Assessing the role of environmental regulations in improving energy efficiency and reducing CO2 emissions: Evidence from the logistics industry. Environmental Impact Assessment Review, 2022. 96: p. 106831.

[25] RehmanM.A., et al., Do diversified export, agriculture, and cleaner energy consumption induce atmospheric pollution in Asia? application of method of moments quantile regression. Frontiers in Environmental Science, 2021: p. 497.

[26] FareedZ., et al., Financial inclusion and the environmental deterioration in Eurozone: the moderating role of innovation activity. Technology in Society, 2022. 69: p. 101961.

[27] ChengC., et al., Heterogeneous impacts of renewable energy and environmental patents on CO2 emission-Evidence from the BRIICS. Science of the total environment, 2019. 668: p. 1328–1338. doi: 10.1016/j.scitotenv.2019.02.063 30846196

[28] CharfeddineL. and KahiaM., Impact of renewable energy consumption and financial development on CO2 emissions and economic growth in the MENA region: a panel vector autoregressive (PVAR) analysis. Renewable energy, 2019. 139: p. 198–213.

[29] SaidiK. and OmriA., The impact of renewable energy on carbon emissions and economic growth in 15 major renewable energy-consuming countries. Environmental research, 2020. 186: p. 109567. doi: 10.1016/j.envres.2020.109567 32361260

[30] AdekoyaO.B., et al., How critical are resource rents, agriculture, growth, and renewable energy to environmental degradation in the resource-rich African countries? The role of institutional quality. Energy Policy, 2022. 164: p. 112888.

[31] GrodzickiT. and JankiewiczM., The impact of renewable energy and urbanization on CO2 emissions in Europe–Spatio-temporal approach. Environmental Development, 2022. 44: p. 100755.

[32] HasnisahA., AzlinaA., and CheC.M.I., The impact of renewable energy consumption on carbon dioxide emissions: Empirical evidence from developing countries in Asia. International Journal of Energy Economics and Policy, 2019. 9(3): p. 135.

[33] AliK., JianguoD., and KirikkaleliD., Modeling the natural resources and financial inclusion on ecological footprint: The role of economic governance institutions. Evidence from ECOWAS economies. Resources Policy, 2022. 79: p. 103115.

[34] SinghA.K., et al., Role of financial inclusion, green innovation, and energy efficiency for environmental performance? Evidence from developed and emerging economies in the lens of sustainable development. Structural Change and Economic Dynamics, 2023. 64: p. 213–224.

[35] LeT.-H., LeH.-C., and Taghizadeh-HesaryF., Does financial inclusion impact CO2 emissions? Evidence from Asia. Finance Research Letters, 2020. 34: p. 101451.

[36] ZaidiS.A.H., HussainM., and ZamanQ.U., Dynamic linkages between financial inclusion and carbon emissions: evidence from selected OECD countries. Resources, Environment and Sustainability, 2021. 4: p. 100022.

[37] AhmadM., et al., Financial inclusion, technological innovations, and environmental quality: Analyzing the role of green openness. Frontiers in Environmental Science, 2022: p. 80.

[38] UsmanM., MakhdumM.S.A., and KousarR., Does financial inclusion, renewable and non-renewable energy utilization accelerate ecological footprints and economic growth? Fresh evidence from 15 highest emitting countries. Sustainable Cities and Society, 2021. 65: p. 102590.

[39] QinL., et al., Does financial inclusion limit carbon dioxide emissions? Analyzing the role of globalization and renewable electricity output. Sustainable Development, 2021. 29(6): p. 1138–1154.

[40] KhanA., et al., Geopolitical risk, economic uncertainty, and militarization: Significant agents of energy consumption and environmental quality. Environmental Impact Assessment Review, 2023. 102: p. 107166.

[41] PataU.K., et al., Militarization of NATO countries sparks climate change? Investigating the moderating role of technological progress and financial development. Journal of Cleaner Production, 2023. 409: p. 137241.

[42] BradfordJ.H. and StonerA.M., The treadmill of destruction in comparative perspective: A panel study of military spending and carbon emissions, 1960–2014. Journal of World-Systems Research, 2017. 23(2): p. 298–325.

[43] SmithC.L. and LengefeldM.R., The Environmental Consequences of Asymmetric War: A Panel Study of Militarism and Carbon Emissions, 2000–2010. Armed Forces & Society, 2020. 46(2): p. 214–237.

[44] JorgensonA.K., ClarkB., and KentorJ., Militarization and the environment: a panel study of carbon dioxide emissions and the ecological footprints of nations, 1970–2000. Global Environmental Politics, 2010. 10(1): p. 7–29.

[45] QayyumU., AnjumS., and SabirS., Armed conflict, militarization and ecological footprint: Empirical evidence from South Asia. Journal of Cleaner Production, 2021. 281: p. 125299.

[46] HansonT., Biodiversity conservation and armed conflict: a warfare ecology perspective. Annals of the New York Academy of Sciences, 2018. 1429(1): p. 50–65. doi: 10.1111/nyas.13689 29683517

[47] BrownV.J., BattleScars: Global Conflicts and Environmental Health. 2004, National Institute of Environmental Health Science.

[48] de BruinS.P., et al., Projecting long-term armed conflict risk: An underappreciated field of inquiry? Global Environmental Change, 2022. 72: p. 102423.

[49] ReuvenyR., Mihalache-O’KeefA.S., and LiQ., The effect of warfare on the environment. Journal of Peace Research, 2010. 47(6): p. 749–761.

[50] PathakS., Ecological footprints of war: An exploratory assessment of the long-term impact of violent conflicts on national biocapacity from 1962–2009. Journal of environmental studies and sciences, 2020. 10(4): p. 380–393.

[51] AhmedZ., et al., Towards environmental sustainability: Do financial risk and external conflicts matter? Journal of Cleaner Production, 2022. 371: p. 133721.

[52] ShahzadU., et al., USAID, official development assistance and counter terrorism efforts: Pre and post 9/11 analysis for South Asia. Socio-Economic Planning Sciences, 2020. 69: p. 100716.

[53] SunC., et al., The impact of socio-economic and fractionalization determinants on terrorism in ESNA. Socio-Economic Planning Sciences, 2022. 79: p. 101138.

[54] BildiriciM. and GokmenogluS.M., The impact of terrorism and FDI on environmental pollution: evidence from Afghanistan, Iraq, Nigeria, Pakistan, Philippines, Syria, Somalia, Thailand and Yemen. Environmental Impact Assessment Review, 2020. 81: p. 106340.

[55] BildiriciM.E., Terrorism, environmental pollution, foreign direct investment (FDI), energy consumption, and economic growth: Evidences from China, India, Israel, and Turkey. Energy & Environment, 2021. 32(1): p. 75–95.

[56] ChishtiM.Z., et al., The asymmetric associations between foreign direct investment inflows, terrorism, CO2 emissions, and economic growth: a tale of two shocks. Environmental Science and Pollution Research, 2021. 28(48): p. 69253–69271. doi: 10.1007/s11356-021-15188-4 34296403

[57] BildiriciM.E., GençS.Y., and CastanhoR.A., Environmental Pollution, Terrorism, and Mortality Rate in China, India, Russia, and Türkiye. Sustainability, 2022. 14(19): p. 12649.

[58] BildiriciM.E., LousadaS., and Yılmaz GençS., Terrorism, Freshwater, and Environmental Pollution: Evidence of Afghanistan, Burkina Faso, Iraq, Arab Republic of Egypt, Cameroon, Mali, Mozambique, Niger, Nigeria, Somalia, Syrian Arab Republic, and Pakistan. Water, 2022. 14(17): p. 2684.

[59] MusaM.S., et al., Effects of tourism, financial development, and renewable energy on environmental performance in EU-28: does institutional quality matter? Environmental science and pollution research, 2021. 28(38): p. 53328–53339. doi: 10.1007/s11356-021-14450-z 34031831

[60] JahangerA., UsmanM., and Balsalobre‐LorenteD., Linking institutional quality to environmental sustainability. Sustainable Development, 2022. 30(6): p. 1749–1765.

[61] EdemeR.K. and GodE.E.T., Interactive Effect of Population Growth and Institutional Quality on Environmental Sustainability in West Africa Region, in Environmental Sustainability, Growth Trajectory and Gender: Contemporary Issues of Developing Economies. 2022, Emerald Publishing Limited. p. 37–49.

[62] MajiI.K., et al., Clean energy, institutional quality and environmental sustainability in sub-Saharan Africa. Cleaner Materials, 2022. 6: p. 100135.

[63] RitiJ.S., ShuY., and KamahM., Institutional quality and environmental sustainability: The role of freedom of press in most freedom of press countries. Environmental Impact Assessment Review, 2021. 91: p. 106656.

[64] ZhouC., WangS., and FengK., Examining the socioeconomic determinants of CO2 emissions in China: A historical and prospective analysis. Resources, Conservation and Recycling, 2018. 130: p. 1–11.

[65] McLeanE.V., et al., Household dependence on solid cooking fuels in Peru: an analysis of environmental and socioeconomic conditions. Global Environmental Change, 2019. 58: p. 101961.

[66] LiuJ.-Y., et al., The importance of socioeconomic conditions in mitigating climate change impacts and achieving Sustainable Development Goals. Environmental Research Letters, 2020. 16(1): p. 014010.

[67] ShimizuT. and KikuchiY., Regional suitability for energy carriers in Japan considering socioeconomic conditions and environmental performance. Journal of Cleaner Production, 2021. 318: p. 128461.

[68] NawazS.M.N. and AlviS., Energy security for socio-economic and environmental sustainability in Pakistan. Heliyon, 2018. 4(10): p. e00854. doi: 10.1016/j.heliyon.2018.e00854 30364534 PMC6197421

[69] KhanI. and HouF., The impact of socio-economic and environmental sustainability on CO2 emissions: a novel framework for thirty IEA countries. Social Indicators Research, 2021. 155(3): p. 1045–1076.

[70] NathanielS.P., YalçinerK., and BekunF.V., Assessing the environmental sustainability corridor: Linking natural resources, renewable energy, human capital, and ecological footprint in BRICS. Resources Policy, 2021. 70: p. 101924.

[71] LiR., WangX., and WangQ., Does renewable energy reduce ecological footprint at the expense of economic growth? An empirical analysis of 120 countries. Journal of Cleaner Production, 2022. 346: p. 131207.

[72] LiuH., et al., A non-linear analysis of the impacts of natural resources and education on environmental quality: Green energy and its role in the future. Resources Policy, 2022. 79: p. 102940.

[73] SharifA., et al., Role of green technology, environmental taxes, and green energy towards sustainable environment: Insights from sovereign Nordic countries by CS-ARDL approach. Gondwana Research, 2023. 117: p. 194–206.

[74] SharifA., MehmoodU., and TiwariS., A step towards sustainable development: role of green energy and environmental innovation. Environment, Development and Sustainability, 2023: p. 1–22.

[75] YeasinM. and PaulR.K., OptiSembleForecasting: optimization-based ensemble forecasting using MCS algorithm and PCA-based error index. The Journal of Supercomputing, 2023: p. 1–30.

[76] BeynonM.J., JonesP., and PickernellD., Evaluating EU-Region level innovation readiness: A longitudinal analysis using principal component analysis and a constellation graph index approach. Journal of Business Research, 2023. 159: p. 113703.

[77] HussainS., et al., Financial inclusion and carbon emissions in Asia: Implications for environmental sustainability. Economic and Political Studies, 2023: p. 1–17.

[78] Leal FilhoW., et al., Commentary-empty promises: why declarations and international cooperation on sustainable development often fail to deliver. International Journal of Sustainable Development & World Ecology, 2022. 29(8): p. 850–857.

[79] SueyoshiT., MoF., and WangD.D., Sustainable development of countries all over the world and the impact of renewable energy. Renewable Energy, 2022. 184: p. 320–331.

[80] CastroG.D.R., FernandezM.C.G., and ColsaA.U., Unleashing the convergence amid digitalization and sustainability towards pursuing the Sustainable Development Goals (SDGs): A holistic review. Journal of Cleaner Production, 2021. 280: p. 122204.

[81] OziliP.K., Theories of financial inclusion, in Uncertainty and challenges in contemporary economic behaviour. 2020, Emerald Publishing Limited. p. 89–115.

[82] LinnerA., et al., Interactions Between SDG 14 (Life Below Water) and SDG 16 (Peace, Justice, and Strong Institutions): A Review of Co-benefits, Synergies, Conflicts, and Trade-Offs. Bridging Peace and Sustainability Amidst Global Transformations, 2023: p. 31–51.

[83] BellK., et al., The necessity of a transformational approach to just transition: defence worker views on decarbonisation, diversification and sustainability. Environmental Politics, 2023: p. 1–21.

[84] AhmedZ., et al., The trade-off between energy consumption, economic growth, militarization, and CO2 emissions: does the treadmill of destruction exist in the modern world? Environmental Science and Pollution Research, 2022. 29(12): p. 18063–18076.34677772 10.1007/s11356-021-17068-3

[85] FanH., et al., How do urbanization and urban agglomeration affect CO2 emissions in South Asia? Testing non-linearity puzzle with dynamic STIRPAT model. Chinese Journal of Urban and Environmental Studies, 2020. 8(01): p. 2050003.

[86] SaqibN., et al., Pollution haven or halo? How European countries leverage FDI, energy, and human capital to alleviate their ecological footprint. Gondwana Research, 2023. 116: p. 136–148.

[87] NchofoungT.N. and AsonguS.A., Effects of infrastructures on environmental quality contingent on trade openness and governance dynamics in Africa. Renewable Energy, 2022. 189: p. 152–163.

[88] UllahA., et al., The dynamic nexus of E-Government, and sustainable development: Moderating role of multi-dimensional regional integration index in Belt and Road partner countries. Technology in Society, 2022. 68: p. 101903.

[89] HuhH.S. and ParkC.Y., A new index of globalisation: Measuring impacts of integration on economic growth and income inequality. The World Economy, 2021. 44(2): p. 409–443.

[90] AdeleyeN. and EboaguC., Evaluation of ICT development and economic growth in Africa. NETNOMICS: Economic Research and Electronic Networking, 2019. 20(1): p. 31–53.

[91] AhmadM., et al., Innovation, foreign direct investment (FDI), and the energy–pollution–growth nexus in OECD region: a simultaneous equation modeling approach. Environmental and Ecological Statistics, 2020. 27(2): p. 203–232.

[92] ArellanoM. and BondS., Some tests of specification for panel data: Monte Carlo evidence and an application to employment equations. The review of economic studies, 1991. 58(2): p. 277–297.

[93] BondS.R. and WindmeijerF., Finite sample inference for GMM estimators in linear panel data models. 2002.

[94] RoodmanD., How to do xtabond2: An introduction to difference and system GMM in Stata. The stata journal, 2009. 9(1): p. 86–136.

[95] BandayU.J. and KocogluM., Modelling simultaneous relationships between human development, energy, and environment: Fresh evidence from panel quantile regression. Journal of the Knowledge Economy, 2023. 14(2): p. 1559–1581.

[96] GujaratiD.N., Linear regression: A mathematical introduction. Vol. 177. 2018: SAGE publications.

[97] AwadA. and WarsameM.H., The poverty-environment nexus in developing countries: evidence from heterogeneous panel causality methods, robust to cross-sectional dependence. Journal of Cleaner Production, 2022. 331: p. 129839.

[98] KoseogluA., YucelA.G., and UlucakR., Green innovation and ecological footprint relationship for a sustainable development: Evidence from top 20 green innovator countries. Sustainable development, 2022. 30(5): p. 976–988.

[99] PaulS.C., RosidM.H.O., and BiswasJ., Impact of Energy and Natural Resources Rent on FDI: An Analysis through POLS, DK, 2SLS and GMM Models. Energy Economics Letters, 2021. 8(2): p. 122–133.

[100] de OliveiraH.V.E. and MoutinhoV., Do renewable, non-renewable energy, carbon emission and KOF globalization influencing economic growth? Evidence from BRICS’countries. Energy Reports, 2022. 8: p. 48–53.

[101] MujtabaA., et al., Symmetric and asymmetric impact of economic growth, capital formation, renewable and non-renewable energy consumption on environment in OECD countries. Renewable and Sustainable Energy Reviews, 2022. 160: p. 112300.

[102] SinghA.K., et al., Role of Financial Inclusion, Green Innovation, and Energy Efficiency for Environmental Performance? Evidence from Developed economies in the lens of Sustainable Development. Structural Change and Economic Dynamics, 2022.

[103] JingpengL., et al., Nonlinear and nonparametric causal relationship between financial inclusion and sustainable environment in South Asia. Environmental Science and Pollution Research, 2023. 30(1): p. 2218–2232. doi: 10.1007/s11356-022-22301-8 35931851

[104] ChangS., ChenB., and SongY., Militarization, renewable energy utilization, and ecological footprints: Evidence from RCEP economies. Journal of Cleaner Production, 2023. 391: p. 136298.

[105] EreghaP.B., VoX.V., and NathanielS.P., Military spending, financial development, and ecological footprint in a developing country: insights from bootstrap causality and Maki cointegration. Environmental Science and Pollution Research, 2022. 29(55): p. 83945–83955. doi: 10.1007/s11356-022-21728-3 35776309

[106] GodefroidtA. and LangerA., How fear drives us apart: Explaining the relationship between terrorism and social trust. Terrorism and Political Violence, 2020. 32(7): p. 1482–1505.

[107] AbidN., et al., Cities trajectories in the digital era: Exploring the impact of technological advancement and institutional quality on environmental and social sustainability. Journal of Cleaner Production, 2022. 377: p. 134378.

[108] AhmadM., et al., Financial development and environmental degradation: do human capital and institutional quality make a difference? Gondwana Research, 2022. 105: p. 299–310.

